RETRACTED

# Construction of Economic Security Early Warning System Based on Cloud Computing and Data Mining

**DOI:** 10.1155/2022/2080840

**Published:** 2022-06-08

**Authors:** Guanghui Yuan, Fei Xie, Huiling Tan

**Affiliations:** ^1^School of Economics and Management, Shanghai University of Political Science and Law, Shanghai 201701, China; ^2^School of Finance, Shanghai University of Finance and Economics, Shanghai 200433, China; ^3^Shanghai Financial Intelligent Engineering Technology Research Center, Shanghai University of Finance and Economics, Shanghai 200433, China; ^4^School of Humanities, Shanghai University of Finance and Economics, Shanghai 200433, China

## Abstract

Economic security is a core theoretical issue in economics. In modern economic conditions, the ups and downs caused by economic instability in any economic system will affect the stability of the financial market, bring huge losses to the economy, and affect the development of the whole national economy. Therefore, research on the regularity of economic security and economic fluctuations is one of the important contents to ensure economic stability and scientific development. Accurate monitoring and forecasting of economic security are an indispensable link in economic system regulation, and it is also an important reference factor for any economic organization to make decisions. This article focuses on the construction of an economic security early warning system as the main research content. It integrates cloud computing and data mining technologies and is supported by CNN-SVM algorithm and designs an early warning model that can adaptively evaluate and warn the economic security state. Experiments show that when the CNN network in the model uses ReLU activation function and SVM uses RBF function, the prediction accuracy can reach 0.98, and the prediction effect is the best. The data set is verified, and the output *Q* province's 2018 economic security early warning comprehensive index is 0.893. The 2019 economic security early warning index is 0.829, which is consistent with the actual situation.

## 1. Introduction

### 1.1. Background Meaning

In today's economic globalization and economic liberalization, economic security is threatened by more risk factors such as the imbalance of national policies and economic structure. Because of the complexity of economic security early warning and monitoring, in most cases, early warning is selected alternately according to some standards of economic crisis monitoring. However, more often, the safety measures taken due to inaccurate prediction may not be in line with the actual situation of economic operation and cannot be adjusted rapidly with the changes of influencing factors. Traditional economic security risk assessment methods are inaccurate and have poor adaptability. The continuous development of cloud computing and big data mining technology has made it possible to construct an adaptive economic security early warning model. The financial systems of various economic organizations and enterprises are gradually becoming informatized, and there have been many financial systems built on the cloud. It is inevitable that it uses network technology, cloud computing, and data mining technology to assist economic security assessment. It is necessary to establish a scientific economic early warning index system and adopt effective data mining methods. It is conducive to the timely adjustment and formulation of economic policies by relevant departments. It can also guide investors to make reasonable investment decisions and can take timely measures to deal with risks and reduce economic losses. It is beneficial to prevent economic risks in advance, reduce economic losses to the lowest limit, make the economic development able to run smoothly, and promote the long-term healthy development of economy. Therefore, the research of this article has very important theoretical value and practical significance.

RETRACTED

### 1.2. Related Work

In the model, the parameters of the economic activities of agricultural and industrial enterprises are characterized by some quantitative and qualitative indicators, which can reflect the level of economic security [1, 2]. The economic security level assessment model in that research does not use too much big data analysis technology and has a narrow scope of application, but its theory can provide help for this article. In the context of the financial management elements selected in 2010 and 2015, the real-time data of that research is poor, and the result analysis may be inaccurate due to data loss. Ruza C. et al. put forward a comprehensive index (CI) to analyze the stability and adaptability of the banking system in developed countries. This indicator does not predict the future behavior of banks but uses it as a tool to assess the overall health of the most important banking system. Taking into account the review of the previous literature, they designed a theoretical framework of flexibility and stability [3]. Trahay F. et al. proposed a data prefetching program, which is mainly for cloud computing dispersed file system. In this prefetching technology, the client basically does not participate in the data prefetching process [4]. The cloud computing distributed solution can better obtain user data, but their research is still insufficient for practical applications. Qian W. et al. obtained the relationship between financial data through fuzzy cognitive map and then inferred and calculated the system crisis value, thus forming a financial crisis early warning algorithm. The financial data of a company is used to verify the effectiveness and feasibility of the algorithm [5]. This method has good predictability and can infer economic security outlook through fuzzy cognitive maps, which has great reference significance for the research of this article. Kang Q. used regression analysis method to make quantitative regression analysis on the influencing factors of various subjects in the financial field on financial security. Based on the economic game theory, big data technology is used to predict the possible risks in the financial field. Finally, an adaptive financial risk assessment scheme is formed [6]. His research is both theoretically and methodologically good, but no applied analysis of actual data has been carried out, and its predictive effect needs to be further verified.

RETRACTED

### 1.3. Innovation

In recent years, the multiclassification algorithms of CNN model and SVM model in machine learning algorithms are widely used in natural language processing and text classification. This article combines the two for economic index forecasting. The innovations of this article are as follows: The first is to construct a system of economic security indicators based on the provincial scale, using a combination of analytic hierarchy process and factor analysis to determine indicator weights; the second is to combine the CNN model and the SVM model to build an early warning model, combining the feature extraction advantages of CNN with the classification advantages of SVM; the third is to use different activation functions for CNN and SVM models to conduct comparative experiments to obtain the best combination model.

## 2. Construction Method of Economic Security Early Warning System Based on Cloud Computing and Data Mining

### 2.1. Cloud Computing and Key Technologies

Cloud computing is to decompose the huge data processing program into countless small programs through the network cloud and then process and analyze these small programs through the system composed of multiple servers to get the results and return to the user. Cloud computing actually represents a new application system organization model and method. From the perspective of information system resources and capability value, it quickly adjusts and adapts the information system architecture according to actual application requirements and service scenarios [7]. From the perspective of architecture, cloud computing provides a more convenient way for enterprise business processing, makes the way of business processing more intelligent, and promotes enterprise transformation; IT also provides a new accounting method for enterprise data accounting and a new IT resource delivery model. It transforms the data center system from centralized equipment operation control to business integration to a “service” platform. It also provides new ideas for the operation of information systems through the transformation of services and at the same time has become a new driving force for information innovation.

RETRACTED

Hadoop is a distributed system infrastructure developed by the Apache Foundation that allows users to develop distributed programs to take full advantage of the power of clusters for high-speed computing and storage without understanding the underlying details of distribution. It is a reliable and scalable open-source distributed computing architecture. It can be used for big data storage and can be used for batch processing in distributed clusters of cross-business and available hardware. The composition of the Hadoop framework is shown in Figure 1. The main four modules are the distributed file system HDFS, the computing framework MapReduce, YARN, and Hadoop Common, and the first two modules are the core modules of the system. The YARN module is used to manage and store data and analyze the resources required by the system when it is running, and Hadoop Common is used to provide the Java libraries and utilities required by the Hadoop module.

HDFS is the core project of the Hadoop project. It has the characteristics of high fault tolerance, high reliability, and high throughput and provides reliable storage for massive data. HDFS uses master/slave devices, as shown in Figure 2. HDFS is a master-slave architecture consisting of node names and a certain number of data nodes. It is usually a machine node, responsible for managing the corresponding storage node. The name node is used to manage names and modify access requests to the client, and the data node is mainly used to store data. HDFS opens the file space, allowing users to store data in file format. Data node also executes instructions for block creation and deletion, as well as block copy node name [8].

MapReduce is a programming model for parallel computation of large data sets (larger than 1TB). With this mode, programmers can easily develop distributed parallel programs without understanding the underlying details of the Hadoop distributed system. Implementing MapReduce on Hadoop has many slave devices connected to a single master node. The master node monitors the slave stations and satisfies resource requirements. After a certain interval, the master node regularly monitors the activities of the slave nodes in the cluster. Hadoop MapReduce processes data on disk through Map and Reduce operations. MapReduce divides the work into two types of tasks, namely, “MapTask” and “ReduceTask,” which help to process large-scale data [9]. The operation process of MapReduce is divided into three phases: Map phase, Shuffle phase, and Reduce phase, as shown in Figure 3.

RETRACTED

### 2.2. Forecasting Model Based on Data Mining Technology

The process of data mining includes data set selection, data set preprocessing, and data mining using certain algorithms to discover hidden useful information. Data mining methods use a large amount of data analysis and find the most valuable law from the massive and redundant data. The models used for prediction in data mining algorithms mainly include regression analysis, regression trees, neural networks, and SVM, all of which belong to supervised learning [10].

#### 2.2.1. Support Vector Machine Regression (SVR) Prediction Model

SVM is a kind of generalized linear classifier for binary classification of data by supervised learning. Its decision boundary is the maximum margin hyperplane of learning samples. The purpose of SVR to construct a classification surface is to minimize the distance between all sample data and the classification surface. Support vector machine regression can reduce the prediction error by appropriate mapping function, and the support vector regression model can add loss function to the classification model to correct the distance [11].

For a training data set, regression is to get the regression function:

(1) $$\begin{array}{c} g\left(y\right)=K\cdot y+a, \end{array}$$

where *K·y* is the inner product of *K* and *y*, and the constraints of the constrained optimization problem are

(2) $$\begin{array}{c} \frac{\text{Min}}{2k\cdot k}+A\sum_{i=1}^{n}\left(\xi_{i}+\xi_{i}^{*}\right),\\ Z_{i}-k\cdot y_{i}+a\leq \varepsilon +\xi_{i},\\ k\cdot y_{i}-z_{i}+a\leq \varepsilon +y_{i}-y_{m}. \end{array}$$

*A* is the penalty factor of the model.

Solving the optimization problem is now converted to a dual problem, and then the kernel function is introduced to solve the maximum constraint value. The model regression equation is

(3) $$\begin{array}{c} g\left(y\right)=\sum_{i=1}^{n}\left(a_{j}-a_{j}^{*}\right)\cdot k\left(y,y_{j}\right)+b. \end{array}$$

#### 2.2.2. Gradient Boosting Decision Tree (GBDT) Algorithm

Boosting enhancement algorithm is a framework algorithm. It extracts sample data to obtain subdata and then uses a weak classification algorithm to train a subset of sample data to generate a set of basic classifiers. Weak classification algorithm is one of the weak classifiers, which can improve the accuracy and reduce the error of the algorithm. The enhanced algorithm can establish a robust ensemble model based on the generalization performance of ultraweak learners, which can be used to improve the classification accuracy of other weak classification algorithms [12].

RETRACTED

Gradient boosting decision tree (GBDT) algorithm belongs to gradient boosting algorithm or classification algorithm and also belongs to ensemble learning. The specific idea is to iteratively generate multiple weak models and then add the prediction results of each weak model and then build the next model on the basis of the original learning model [13]. GBDT can be seen as an additive model composed of W trees:

(4) $$\begin{array}{c} {\hat{y}}_{i}=\sum_{w-1}^{W}f_{w}\left(x_{i}\right),\;f_{w}\in F. \end{array}$$

The objective function of the algorithm addition model is defined as

(5) $$\begin{array}{c} O=\sum_{i-1}^{m}\gamma \left(y_{i},{\hat{y}}_{i}\right). \end{array}$$

The calculation process using the forward distribution algorithm is as follows:

(6) $$\begin{array}{c} {\hat{y}}_{i}^{0}=0,\\ {\hat{y}}_{i}^{1}=f_{1}\left(x_{i}\right)={\hat{y}}_{i}^{0}+f_{1}\left(x_{i}\right),\\ {\hat{y}}_{i}^{2}=f_{1}\left(x_{i}\right)+f_{2}\left(x_{i}\right)={\hat{y}}_{i}^{1}+f_{2}\left(x_{i}\right),\\ {\hat{y}}_{i}^{s}=\sum_{w-1}^{s}f_{w}\left(x_{i}\right)={\hat{y}}_{i}^{s-1}+f_{s}\left(x_{i}\right), \end{array}$$

and, in step *S*, the model's prediction of *x* is

(7) $$\begin{array}{c} {\hat{y}}_{i}^{s}={\hat{y}}_{i}^{s-1}+f_{s}\left(x_{i}\right). \end{array}$$

In the above formula, *f*_*s*_(*x*_*i*_) is the function of the decision tree to be learned by the algorithm in this round. At this time, the objective function can be written as

(8) $$\begin{array}{c} O^{s}=\sum_{i-1}^{m}\gamma \left(y_{i},{\hat{y}}_{i}^{s}\right)\sum_{i-1}^{m}\gamma \left(y_{i},{\hat{y}}_{i}^{s-1}+f_{s}\left(x_{i}\right)\right). \end{array}$$

Adding the square error of the loss function yields

(9) $$\begin{array}{c} \gamma \left(y_{i},{\hat{y}}_{i}^{s}\right)={\left(y_{i}-{\hat{y}}_{i}^{s}\right)}^{2}. \end{array}$$

In the end,

(10) $$\begin{array}{c} \gamma \left(y_{i},{\hat{y}}_{i}^{s-1}+f_{s}\left(x_{i}\right)\right)\left(\right)={\left(y_{i}-{\hat{y}}_{i}^{s}-f_{s}\left(x_{i}\right)\right)}^{2}={\left(r-f_{s}\left(x_{i}\right)\right)}^{2},\\ R=y_{i}-{\hat{y}}_{i}^{s-1}. \end{array}$$

*r* is the residual, and the process of GBDT iteration is the process of fitting the residual.

Using the publicly unbalanced data set, the GBDT and logistic regression algorithm were used for comparative experiments, and then the ROC curve was taken to measure the classification model learned by the two algorithms on the unbalanced data set. The result is shown in Figure 4.

RETRACTED

#### 2.2.3. Early Warning Model Based on Convolutional Neural Network and Support Vector Machine (CNN-SVM)

CNN model is a deep feedforward artificial neural network. Its structure can also be feature extraction and processing (prediction) module. The feature extraction module is mainly composed of continuous convolution and pooling layers, and the processing (prediction) module is mainly composed of fully connected layers. However, a major disadvantage of CNN is overfitting and local overoptimization in which overfitting refers to the analysis results that are too closely or precisely corresponding to a particular data set and therefore may not be able to fit other data or reliably predict future observations [14]. Then the nonlinear SVM model can effectively avoid the disadvantages of CNN by introducing relaxation variables and finally get the optimal solution. To sum up, this paper chooses to combine the advantages of CNN and SVM, that is, to replace the fully connected layer of CNN model with nonlinear SVM classifier to build a combined model.

The CNN-SVM combined model is shown in Figure 5. The concrete steps of the model operation are as follows: First, preprocess the sample data; second, set model parameters and initialize; third, transform the panel data of economic training set into matrix. Input it into CNN model as input vector, and import the feature vector output by CNN into SVM training model parameters; fourth, output the test set data into a matrix, and then introduce it into the trained model to get the final prediction result, and calculate the judgment coefficient with the actual warning level [15].

### 2.3. Risk Early Warning Assessment Method

#### 2.3.1. Analytic Hierarchy Process (AHP)

The analytic hierarchy process (AHP) is an analysis method proposed by American Journal of Operations Research to solve multiobjective decision-making problems. The analytic hierarchy process (AHP) is a decision-making method that disintegrates the elements always related to decision-making into the levels of objectives, criteria, and schemes and makes qualitative and quantitative analysis on this basis. It is a combination of quantitative analysis and qualitative analysis. The analytic hierarchy process (AHP) decomposes complex issues into different hierarchical structures according to the superiority relationship. It then compares the importance of the two factors and then ranks the importance of each factor [16].

The specific steps of the analytic hierarchy process are as follows: First, a systematic hierarchical structure model is established, which is generally divided into several levels according to the subordination of factors. Second, a judgment matrix for pairwise comparison is constructed to determine the number of lower-level factors determined by the influencing factors and the ranking of their weights and determine these weights. Generally, the 9-scale method is used for assignment, as shown in Table 1.

RETRACTED

Third, according to certain influence criteria, the weight of control factors is calculated, the consistency of judgment matrix is checked, the judgment matrix that does not conform to the consistency is corrected, and the weight of each factor in the total objective factor is calculated.

#### 2.3.2. Factor Analysis (FA)

Factor analysis uses multiple factors to describe the relationship between multiple indicators or factors. It finds the same factors in the variable search process and classifies them into the same category. That is, the variable becomes a factor, and fewer factors reflect most of the information of the original data [17].

Factor analysis expresses variables as linear combinations of factors in the form of regression equations:

(11) $$\begin{array}{c} y_{1}=a_{11}f_{1}+a_{12}f_{2}+\cdots +a_{1n}f_{n}+\varepsilon_{1},\\ y_{2}=a_{21}f_{1}+a_{22}f_{2}+\cdots +a_{2n}f_{n}+\varepsilon_{2},\\ y_{k}=ya_{k1}f_{1}+a_{k2}f_{2}+\cdots +a_{kn}f_{n}+\varepsilon_{k},\\ y=\left(y_{1},y_{2},\ldots ,y_{k}\right), \end{array}$$

where *a*_*ii*_ is the load factor and *f* is the common factor of *y*. The matrix form is

(12) $$\begin{array}{c} y=Af+\varepsilon , \end{array}$$

and factor analysis is a combination of variables representing common factors. Because the factor can reflect the relationship between the original variables, sometimes the common factor needs to be converted into a linear combination, that is, the factor score:

(13) $$\begin{array}{c} f_{i}=b_{i1}y_{1}+b_{i2}y_{2}+\cdots +b_{ik}y_{k};\;\left(i=1,2,\ldots ,n\right). \end{array}$$

#### 2.3.3. Fuzzy Comprehensive Evaluation (FCE) Method

Fuzzy comprehensive evaluation is a comprehensive evaluation theory that combines fuzzy mathematics with decision-making methods. It uses the method of fuzzy mathematics to transform the qualitative factors in the evaluation index into quantitative factors, which is convenient for sorting the target problems. This method can effectively solve the problem of ambiguity in the evaluation process. For example, the affiliation of some indicators is fuzzy, and experts are not clear enough about the importance of some indicators [18]. The fuzzy comprehensive evaluation method has obvious advantages, the mathematical model is simple, and it is easy to solve problems with many indicators and complex levels. However, the method itself has certain limitations, such as complex calculation process and easy loss of information.

RETRACTED

The steps of safety early warning assessment based on fuzzy theory are as follows. The first is to build a risk index evaluation system. In this step, it is necessary to summarize and classify the various influencing factors that may affect economic security and establish a target hierarchical structure; the second is that it standardizes the original data, which is convenient for quantitative calculation of the results, but, generally speaking, there are different metrics for different indicators; finally, it uses the normalization formula for comprehensive evaluation, starting from the bottom of the indicator system and finally getting the overall target evaluation value, and the larger the value, the better the subject's situation.

### 2.4. Construction of the Economic Security Risk Early Warning Model

#### 2.4.1. Basis for the Construction of Indicators

Economic crises often have precursors, which are reflected in abnormal changes in some economic factors [19]. Therefore, it is necessary to establish an indicator system. The economic safety index system is the monitoring and measurement of system safety. Different from macroeconomics, the research scope of this article is mainly the early warning of provincial economic security. When studying provincial economic security, we must pay attention to the key factors of provincial economic risks. Provincial economic risk has its own particularity and difference; the study of its particularity and difference is helpful for local governments to formulate the correct strategy of provincial economic development.

The basic basis for constructing the indicator system is as follows. The first is to combine comprehensiveness and focus, and the index system should cover a wide range, involving all aspects of economic security. At the same time, it is necessary to screen out indicators that can reflect the degree of economic risk; the second is to ensure operability and practicality. The selected indicators must be clear, and the data can be obtained and authoritative, while avoiding the use of indicators that cannot be quantified; the third is to focus on hierarchy and comprehensiveness. Each upper-level index has a corresponding lower-level index, and the function and category of each goal are clearly defined [20].

#### 2.4.2. Establishment of Indicator System

After analysis, this paper adopts top-down weight assignment in the process of determining indicators. It first uses the analytic hierarchy process to assign weights to the second-level indicators, and the weight of the third-level index is determined by factor analysis. This article monitors economic security data from the objective of measuring the continued stability of the economy, the balance of government revenue and expenditure, the rationality of the industrial structure, and the sustainability of the economy. In summary, the secondary indicators selected in this article are economic growth, fiscal finance, industrial structure, ecosystem, and consumption structure. The primary and secondary indicators are described by multiple qualitative and quantitative indicators, and the established indicator system is shown in Table 2.

RETRACTED

From this, we get the comprehensive early warning index on the economic security of the province:

(14) $$\begin{array}{c} I=\frac{\sum_{i=1}^{n}x_{j}w_{j}}{\sum_{i=1}^{n}w_{j}}. \end{array}$$

In the above formula, *n* is the number of indexes, w_*j*_ is the weight of the *j*-th index, and 1 is the value of the *j*-th index for normalization processing. The early warning results are classified according to the comprehensive early warning index, and the specific description is shown in Table 3. Among them, no early warning and light early warning are considered to be safe in the economic state, and medium early warning and severe early warning are all considered to be risky in economic security.

## 3. Empirical Analysis of Economic Security Early Warning System Based on CNN-SVM

### 3.1. CNN-SVM Algorithm Implementation

#### 3.1.1. Experimental Environment Construction

The Hadoop operating environment is generally Linux. However, due to the limitation of the experimental environment, it is also convenient for research and experiment. This experiment uses Windows to install the virtual server. The virtual server installs the Linux system to implement Hadoop in the Linux environment. In this experiment, it uses VMware Workstation Pro virtual machine to create eight virtual servers to build a Hadoop cluster.

#### 3.1.2. Source of Experimental Data Set

This article mainly focuses on the research of provincial economic security early warning and chooses Chinese Q province as the research object. The data set comes from the Wind Economic Database, which integrates massive global macro and industry statistics. The experimental data are divided into two categories. One is panel data, which is used for training and testing; the other part is the actual warning level data, which is used for comparative analysis with the model warning results. In order to enhance the applicability of the model, the sample is randomly divided into a training set and a test set. The ratio is 6 : 4, and the random division is performed ten times to obtain ten data sets. It inputs the data set into CNN-SVM combined model, finally obtains the accuracy of observation classification, and averages ten groups of early warning indicators to obtain the final economic security early warning level. The monthly data of Q province from January 2016 to January 2020 were reselected from the Wind database, with a total of 48 samples.

RETRACTED

#### 3.1.3. CNN-SVM Model Parameter Setting

The CNN model needs to set the size and number of convolution kernels of the convolutional layer, pooling layer, convolutional layer, and pooling layer. The specific settings are shown in Table 4. CNN's convolution and pooling layers are set to 3 layers. The convolution sums of convolution layer and pool layer are 5*∗*5 and 3*∗*3, respectively. The initial value of CNN model iteration number is set to 100, and SVM adopts one-to-many method.

### 3.2. CNN-SVM Model Economic Security Prediction Accuracy Analysis

#### 3.2.1. Accuracy Analysis of the CNN Model

The activation function in CNN can be ReLU function or tan*h* function. It uses the ten data sets mentioned above for experiments. CNN uses ReLU and tan*h* functions to test, respectively, to calculate the coincidence accuracy between the actual values of the predicted range. The experiment is shown in Figure 6. It can be concluded that the exact values of CNN model under the two activation functions are not much different. In order to further distinguish the difference between the ReLU function and the tan*h* function to predict the exact value of the CNN convolutional neural network, this paper also calculates the average value of the abovementioned experimental step structure. The results are as follows: When CNN-ReLU function is used, the prediction accuracy is 0.62, and when tan*h* function is introduced, the prediction accuracy is 0.609. To sum up, among the two functions, CNN's prediction performance with ReLU is the best.

#### 3.2.2. CNN-SVM Model Prediction Accuracy Analysis

*(1) The Influence of Activation Function on Model Accuracy*. CNN uses ReLU and SVM uses Polynomial (Poly), LR, RBF, and sigmoid functions, respectively, to experiment with data sets, and the final accuracy results are shown in Figure 7. From the figure, it can be seen that CNN-SVM model performs well under four activation functions. However, when RBF function is used, the accuracy of CNN-SVM combined model is relatively good. SVM uses Poly, LR, RBF, and sigmoid functions to predict the accuracy of ten groups of experimental data. The average prediction accuracy is 0.913, 0.925, 0.983, and 0.95.

When CNN model uses tan*h* function and SVM uses Poly, LR, RBF, and sigmoid functions, respectively, experiments are carried out on data sets, and the final accuracy results are shown in Figure 8. When SVM uses Poly, LR, RBF, and sigmoid functions, the average accuracy of 10 groups of experimental data is predicted to be 0.8599, 0.907, 0.964, and 0.92. In this case, that is, CNN uses tan*h* function and SVM uses RBF function, the accuracy of CNN-SVM combined model is relatively high.

*(2) The Relationship between Iteration Times and Model Prediction*. For the two models with the highest prediction accuracy in the previous test model, namely, (CNN—ReLU; SVM—RBF) model and (CNN—tan*h*; SVM—RBF) model, the iteration times of these two models are set to 100, 200, 600, and 1200, respectively, and experiments are carried out. The average values of the test results of ten groups of data values are also calculated, and the influence of different iterations on the model accuracy is observed. The result is shown in Figure 9.

RETRACTED

In figure (A), it can be seen that when the number of iterations is 1200, the accuracy value is the highest, the prediction accuracy values of the ten data sets are higher than those in the other iteration times, and the average accuracy can reach 0.991; in figure (B), the model prediction accuracy of different iteration times is not much different. On the whole, when CNN uses ReLU function to activate, SVM applies RBF function, and the number of iterations is 1200, the prediction accuracy is the highest, which is 0.991.

### 3.3. Effect Analysis of Economic Security Early Warning System Based on CNN-SVM Algorithm

Based on the above experiments, the optimal predictive value model has been obtained. This section will conduct an empirical analysis of its early warning effect. It uses Q province's data from 2018 to 2019 as a sample set for early warning testing. It compares the test results with the actual warning levels to verify the validity of the optimal model proposed in this experiment.  Figure 10 shows the output results of the five first-level indicator systems in the indicator system of the economic security early warning system. The five indicators of economic growth, finance, industrial structure, ecosystem, and consumption structure are represented by letters *A* to *E* in the figure, and the comprehensive early warning index is represented by *I*. Under the CNN-SVM economic security early warning model, the output Q province's 2018 comprehensive economic security early warning index is 0.893, and the 2019 economic security early warning index is 0.829. From the classification of the economic security early warning index system designed in our study, the economic early warning level of Q province in 2018 is at a light early warning (IV). Relatively speaking, the economy is in a relatively safe state, and the economic warning level in 2019 is medium warning (III), and economic security is in a state of risk. The forecast result of the early warning is consistent with the early warning grade given in Wind economic database, which shows that the economic security early warning system designed in this paper based on the CNN-SVM algorithm has a higher accuracy in predicting economic security.

RETRACTED

## 4. Discussion

This article summarizes the relevant theories and research content of cloud computing, data mining, and economic security index systems. Based on the above-mentioned theory, it uses analytic hierarchy process and factor analysis to construct a provincial economic security index system. An adaptive provincial economic security early warning model based on CNN-SVM combined algorithm is proposed, and the combination of optimal activation function and iteration times of CNN and SVM in the model is studied. The results show that when CNN uses ReLU function, SVM uses Gaussian RBF kernel function, and the number of iterations is 1200, the prediction accuracy of the model is the best. Then it uses the model to conduct empirical analysis on the data set, and the results confirm that the results of the model's early warning of provincial economic security are highly consistent with the actual situation, and the model is effective. The economic security early warning system constructed in this paper can help the formulation of economic policies and promote the smooth operation of the economy.

## 5. Conclusions

According to the research results related to the index system of economic monitoring system, it is found that most of the research is still in the stage of qualitative analysis, and, comparatively speaking, quantitative analysis is less. This article is based on cloud computing and big data to build an adaptive economic security early warning system that can combine quantitative analysis and qualitative analysis. The economic security monitoring and early warning model based on convolutional neural network and support vector machine is constructed in this paper. It combines the powerful feature extraction capabilities of convolutional neural networks with the stable classification capabilities of support vector machines, which can effectively process various economic-related data. The experimental results also verify that the economic security early warning model constructed in this paper has a good performance. It has high accuracy in predicting data sets and can accurately describe economic operation conditions, and the early warning results are consistent with actual scenarios and have good applicability. Since the economic security early warning system studied in this paper is only suitable for the provincial economy and not suitable for the prediction of macroeconomic security risks, it is hoped that the future research can focus on macroeconomic security risks.

RETRACTED

## Figures and Tables

**Figure 1:** Hadoop framework system.

**Figure 2:** HDFS workflow.

**Figure 3:** MapReduce data processing flow.

**Figure 4:** ROC curve comparison of LR and GBDT algorithm results.

**Figure 5:** CNN-SVM model structure.

**Figure 6:** CNN prediction accuracy under different activation functions.

**Figure 7:** CNN-SVM prediction accuracy. (a) Poly. (b) LR. (c) RBF. (d) Sigmoid.

**Figure 8:** CNN-SVM prediction accuracy (CNN_tan*h*). (a) Poly. (b) LR. (c) RBF. (d) Sigmoid.

**Figure 9:** Selection of optimal model and optimal number of iterations.

**Figure 10:** 2018-2019 Q province's economic security warning results.

**Table 1:** The meaning of scaling method.

Degree of importance of “A is more important than B”	Score value	Intermediate value
0	1	2 4 6 8
1	3	
2	5	
3	7	
4	9	

**Table 2:** Provincial economic security index system.

Provincial economic security			
Primary index	Secondary index	Index nature	Weight
Economic growth (A) 0.2157	A1: GDP growth per capita	+	0.2146
	A2: growth rate of fixed assets	+	0.2243
	A3: investment in infrastructure	+	0.2172
	A4: import and export volume	+	0.1938
	A5: dependence on foreign trade	+	0.1501

Finance (B) 0.2011	B1: total revenue and expenditure	+	0.1766
	B2: per capita fiscal revenue	+	0.1515
	B3: per capita financial expenditure	+	0.1645
	B4: tax per capita	+	0.1689
	B5: per capita disposable income of urban households	+	0.1681
	B6: deposit loan ratio of provincial banks	+	0.1704

Industrial structure (C) 0.2034	C1: proportion of tertiary industry	+	0.2045
	C2: proportion of industrial output value	+	0.2178
	C3: average wage level	+	0.1872
	C4: proportion of enterprise scientific research expenses	+	0.1927
	C5: actually utilized foreign capital	+	0.1978

Ecosystem (D) 0.1821	D1: forest coverage	+	0.2547
	D2: total wastewater discharge	−	0.2519
	D3: output of solid waste	−	0.2465
	D4: total dust emission	−	0.2469

Consumption structure (E) 0.1977	E1: retail sales of social consumer goods	+	0.3527
	E2: consumption level of urban residents	+	0.3034
	E3: consumer price index	+	0.3439

**Table 3:** Delineation of warning levels.

*I* value	Early warning level	Economic operation state
0.90 ≤ *I* ≤ 1	V	No warning
0.85 ≤ *I* ≤ 0.90	IV	Light warning
0.65 ≤ *I* ≤ 0.85	III	Moderate warning
0.45 ≤ *I* ≤ 0.65	II	Heavy warning
0 ≤ *I* ≤ 0.45	I	Giant warning

**Table 4:** Convolutional neural network structure.

	Enter figure size	Convolution kernel size	Output figure size
Convolution layer 1	16 × 16	5 × 5	16 × 16
Pool layer 1	16 × 16	3 × 3	8 × 8
Convolution layer 2	8 × 8	5 × 5	8 × 8
Pool layer 2	8 × 8	3 × 3	4 × 4
Full connection layer	16 × 16 × 4 × 4	—	256

RETRACTED

## Data Availability

No data were used to support this study.
